The article "Therapeutic Implications of Some Natural Products for Neuroimmune Diseases: A Narrative of Clinical Studies Review" was published in 2023. Journal: Evid Based Complement Alternat Med.

# Therapeutic Implications of Some Natural Products for Neuroimmune Diseases: A Narrative of Clinical Studies Review

**DOI:** 10.1155/2023/5583996

**Published:** 2023-04-13

**Authors:** Gayathri Wijeweera, Nalaka Wijekoon, Lakmal Gonawala, Yoonus Imran, Chandra Mohan, K. Ranil D. De Silva

**Affiliations:** ^1^Institute for Combinatorial Advanced Research and Education (KDU-CARE), General Sir John Kotelawala Defense University, Sri Lanka; ^2^Interdisciplinary Centre for Innovation in Biotechnology and Neurosciences, Faculty of Medical Sciences, University of Sri Jayewardenepura, Sri Lanka; ^3^Department of Cellular Neuroscience, Faculty of Health, Medicine & Life Sciences, Maastricht University, Maastricht, Netherlands; ^4^Department of Biomedical Engineering, University of Houston, Houston, TX, USA

## Abstract

Neuroimmune diseases are a group of disorders that occur due to the dysregulation of both the nervous and immune systems, and these illnesses impact tens of millions of people worldwide. However, patients who suffer from these debilitating conditions have very few FDA-approved treatment options. Neuroimmune crosstalk is important for controlling the immune system both centrally and peripherally to maintain tissue homeostasis. This review aims to provide readers with information on how natural products modulate neuroimmune crosstalk and the therapeutic implications of natural products, including curcumin, epigallocatechin-3-gallate (EGCG), ginkgo special extract, ashwagandha, *Centella asiatica, Bacopa monnieri,* ginseng, and cannabis to mitigate the progression of neuroimmune diseases, such as Alzheimer's disease, multiple sclerosis, amyotrophic lateral sclerosis, Parkinson's disease, depression, and anxiety disorders. The majority of the natural products based clinical studies mentioned in this study have yielded positive results. To achieve the expected results from natural products based clinical studies, researchers should focus on enhancing bioavailability and determining the synergistic mechanisms of herbal compounds and extracts, which will lead to the discovery of more effective phytomedicines while averting the probable negative effects of natural product extracts. Therefore, future studies developing nutraceuticals to mitigate neuroimmune diseases that incorporate phytochemicals to produce synergistic effects must analyse efficacy, bioavailability, gut-brain axis function safety, chemical modifications, and encapsulation with nanoparticles.

## 1. Introduction

Neuroimmune disorders are multifactorial and include neuroinfectious, autoimmune, paraneoplastic, neurodegenerative, and neuropsychiatric conditions that are primarily characterized by inflammatory responses in the central nervous system (CNS). Even though neuroimmune disorders predominantly manifest as an exaggerated immune response, the underlying pathogenesis involves different immunological mechanisms such as those that are cell-mediated, humoral mediated, or triggered by infection, which is characterized by genetically defined mechanisms for each disorder [1].

The article "Therapeutic Implications of Some Natural Products for Neuroimmune Diseases: A Narrative of Clinical Studies Review" was published in 2023. Journal: Evid Based Complement Alternat Med.

Neuroinflammation is a hallmark responsible for the occurrence of neurodegenerative conditions, including Alzheimer's disease (AD), Parkinson's disease (PD), amyotrophic lateral sclerosis (ALS), Huntington's disease (HD), and multiple sclerosis (MS) [2]. T and B lymphocytes, as well as inflammatory cells in the nervous system such as microglia, oligodendrocytes, and astrocytes, are stimulated by the activation of numerous immune cascades, which play a key role in neuroinflammation and inflammatory cytokines. The activated immune cascade disrupts the blood-brain barrier (BBB) and blood-nerve barrier (BNB), allowing inflammatory cells to infiltrate the nervous system further and the development of neuroimmune disorders. The activation of the various immune cascades stimulates T and B lymphocytes and inflammatory cells in the nervous system, such as microglia, oligodendrocytes, and astrocytes, and plays a pivotal role in neuroinflammation and inflammatory cytokines. The activated immune cascade causes disruption of the BBB and BNB, which allows additional infiltration of inflammatory cells into the nervous system and the development of neuroimmune diseases [3–5].

ALS is a known neurodegenerative disease with a poor prognosis, with few United States Food and Drug Administration (FDA) approved disease-modifying drugs that produce only minimal survival benefits [6]. Studies have estimated that approximately 35 million people worldwide are suffering from the debilitating effects of AD, yet only one recently FDA-approved drug is available to mitigate disease progression [7]. Although approved immunomodulatory therapeutic modalities for MS are available, these drugs have limited efficacy in preventing the transition to the progressive phase of MS, and severe adverse effects have become a major issue with these disease-modifying drugs [8]. The scenario for PD is no exception, as there are limited available therapeutic options to treat PD, and these therapies do not alter the nondopamine-dependent features of PD, especially cognitive impairment [9]. Patients suffering from the aforementioned incurable and debilitating neuroimmune diseases have devastating lifelong functional, physical, and mental disabilities. Additionally, they may have to undergo very expensive, therapeutic interventions that are unaffordable for many, thus creating a great economic burden on their families, especially in developing countries [1]. Several preclinical investigations have found that natural products and their bioactive components can protect against neuroimmune disorders. Therefore, alternative drug discovery based on authentic natural products has the potential to improve the quality of life of patients with neuroimmune diseases by ameliorating disease progression and reducing comorbidities [1, 10, 11].

The article "Therapeutic Implications of Some Natural Products for Neuroimmune Diseases: A Narrative of Clinical Studies Review" was published in 2023. Journal: Evid Based Complement Alternat Med.

The authors aim to provide a review of the existing clinical studies that utilised natural products in South Asia targeted at neuroimmune diseases. Moreover, this review suggests some solutions for enhancing the bioavailability of natural products by optimizing the appropriate dosage, synergetic effects of phytochemicals, chemical modifications, and encapsulation with nanoparticles.

## 2. Review Methodology

The review process was divided into three major steps: title, abstract, and content screening. The previous South Asian natural products studies on neuroimmune disease are reviewed in this article. Articles were searched in databases including PubMed, Medline, Scopus, Embase, and Springer. The search was based on the key words: neuroimmune diseases, neuroimmune crosstalk, and South Asian natural products where a total of 3024 publications were identified.

All the titles were screened, and 1578 documents were downloaded for abstract screening. The inclusion criteria were having the key words “South Asian natural products” and “neuroimmune diseases.” After the abstract screening, a total of 333 articles out of 1578 that met the inclusion criteriawere retained. Finally, full texts of all 333 retained documents were critically assessed using the same inclusion/exclusion criteria as the abstract screening, leaving 105 papers to be included in this review. The review methodology has been summarised in Figure 1.

### 2.1. Neuroimmune Crosstalk in Neuroimmune Diseases

According to Deczkowska and Shwartz, “Immune cells patrol the immune-privileged CNS and support its function”; thus, the modulation of bidirectional neuroimmune crosstalk will open up possibilities to fight against neurological diseases [12, 13]. Although the CNS is comparatively isolated from the peripheral immune system, glial cells play a major anti-inflammatory and neuroprotective role by upregulating anti-inflammatory processes to protect the CNS from stress and noxious pathogens, hence regulating homeostasis [14]. On the other hand, exorbitant or tedious glial activation leads to neuroinflammation and subsequently neurodegeneration [15, 16]. Intriguingly, inflammatory mediators, such as cytokines, chemokines, and cytotoxic molecules, trigger astrocytes to induce secondary inflammatory factors to stimulate a neuroinflammatory cascade [17, 18] (Figure 2).

The article "Therapeutic Implications of Some Natural Products for Neuroimmune Diseases: A Narrative of Clinical Studies Review" was published in 2023. Journal: Evid Based Complement Alternat Med.

Even though the adaptive response from the acute inflammatory response is beneficial to defending against pathogens, chronic neuroinflammation causes tissue destruction and neuronal dysfunction [19]. The underlying molecular mechanisms have been demonstrated by *in vitro* studies, including the upregulation of peroxisome proliferator-activated receptor gamma (PPAR*γ*) and the downregulation of the nuclear factor kappa B (NF-*κ*B) pathway [20, 21]. This leads to inhibition of the activation of microglia, thus diminishing the generation of proinflammatory cytokines and reducing reactive oxygen species (ROS) production via suppression of the Janus kinase 2/signal transducer and activator of transcription 3 (JAK2/STAT3) pathway [22, 23]. Due to the ability of microglia to regulate neuroinflammation, the homeostatic proteins of the microglia have been considered drug targets by modulating signaling pathways such as JAK/STAT and NF-*κ*B [24]. The metabolite of cinnamon and sodium benzoate (NaB) has been shown to reduce glial inflammation, upregulate Tregs via reduction of nitric oxide (NO) inhibition, suppress T helper 17 (Th17) cells and Type 1 T helper (Th1) cells, inhibit inflammatory infiltration, restore the integrity of the BBB, and protect myelin in mouse models of MS [25, 26]. The immunomodulatory properties of NaB may be used against a variety of neuroinflammatory disorders, including MS, as a primary or adjunct therapy [27]. This reduces redox imbalance, oxidative stress, and neuroinflammation, hence combating neuronal damage in neurodegenerative diseases. Prior studies have suggested that the activated, polarized M1 (proinflammatory macrophage) phenotype can be used as a therapeutic target of natural products to treat neurodegenerative diseases [24, 28].

There is a clinical necessity to identify novel compounds to mitigate or treat the diseases associated with neuroimmune communication to reduce the negative effects of microglia and inflammatory cytokines. As summarized in Table 1, natural products may potentially be used as immune modulators to treat neuroimmunological disorders due to their ability to participate in numerous functions of adaptive/innate immunity. In this scenario, natural products and their bioactive compounds, such as curcumin, epigallocatechin-3-gallate (EGCG), ginkgo special extract, ashwagandha, *Centella asiatica, Bacopa monnieri,* ginseng, and cannabis can be used as protective agents against neuronal damage caused by inflammation and oxidative stress [24, 28].

The article "Therapeutic Implications of Some Natural Products for Neuroimmune Diseases: A Narrative of Clinical Studies Review" was published in 2023. Journal: Evid Based Complement Alternat Med.

### 2.2. Curcumin

Curcumin is a yellow-coloured spice that comes from the *Curcuma longa* plant and is widely used in India and Sri Lanka [45]. Curcumin is a lipophilic phenolic diferuloylmethane that has been shown to inhibit a variety of transcription factors, cytokines, protein kinases, interleukins, and enzymes linked to inflammation, making it a potential therapeutic option for neuroimmune diseases such as MS, PD, AD, and ALS [46–48]. Despite multiple encouraging outcomes from *in vivo* and *in vitro* investigations, similar progress in human trials against AD with a 24-week study of a daily dosage of 2 grams or 4 grams of oral Curcumin C3 Complex [32] has not been made. Curcumin's limited bioavailability and solubility likely limit its capacity to reach significant concentrations in the CNS to provide benefit [32]. Curcumin is also poorly absorbed when taken orally, and it undergoes hepatic conjugation, resulting in the generation of biologically inactive metabolites [31], Future research should be designed to optimize curcumin's therapeutic effectiveness. Clinical research comparing the bioavailability of curcumin and piperine, an inhibitor of hepatic and intestinal glucuronidation, revealed that the bioavailability of curcumin rose when piperine was consumed simultaneously, which could explain the reported increase in curcumin activity [45]. Dolati et al. [44] found that supplementing with nanocurcumin for six months can drastically reduce the mRNA expression and secretion levels of proinflammatory cytokines and transcription factors in MS patients. As a result, nanocurcumin could be administered to alleviate MS symptoms.

Polyherbal extracts will be a superior choice for increasing curcumin bioavailability and thus improving its therapeutic efficacy by altering hepatic and intestinal metabolic enzymes and transporters. Chico et al. [31] investigated the efficacy of oral supplementation of Brainoil, a nutraceutical curcumin-based compound, consisting of curcumin (600 mg), 100 mg of Coenzyme Q10, 300 mg of *Bacopa monnieri*, and 250 mg of *Withania somnifera* and *Centella asiatica*. Moreover, Coenzyme Q10 is a potent antioxidant that acts to enhance mitochondrial activity and addition of piperine (1 mg of *Piper nigrum*) to enhance bioavailability. Following 6 months on clinical parameters (Table 1) and biochemical markers in ALS patients found that treatment with curcumin modifies lactate production profile during muscular exercise suggesting improvement in mitochondrial function aerobic metabolism and oxidative damage thus slowing down the disease progression [31].

The exploitation of the synergistic mechanisms of herbal compounds will lead to the discovery of more accomplishable phytomedicines that can avert the probable negative effects of single compounds. It is necessary to conduct human studies to identify possible compounds that could act synergistically with curcumin to enhance its bioavailability and activity [49].

The article "Therapeutic Implications of Some Natural Products for Neuroimmune Diseases: A Narrative of Clinical Studies Review" was published in 2023. Journal: Evid Based Complement Alternat Med.

### 2.3. Epicatechin Gallate (EG) and Epigallocatechin-3-Gallate (EGCG)

Catechins are antioxidants that can be found in fruits such as apples, cherries, apricots, strawberries, and blackberries, as well as in beverages such as black tea and green tea. Its anti-inflammatory and neuroprotective properties could open up new avenues for treating neuroimmune diseases [50]. In a phase 1 clinical trial to investigate the efficacy of EGCG in individuals with MS, 800 mg of polyphenon E failed to restore N-acetyl aspartate (NAA) levels and resulted in increased liver enzyme levels in the participants (Table 1) [39]. To estimate the toxic dosage and bioavailability of EGCG, more clinical investigations are needed. Factors that reduce catechin concentration and inactivation, such as hard water with high Ca2+ and Mg2+ concentrations or even drinking milk with EGCG, should be considered [51]. The intake of EGCG in combination with other dietary components, which modify the context of EGCG before absorption and alter its biological response, has a direct impact on its absorption and stability.

According to Naumovski et al. [52], systemic absorption of EGCG given in capsules without food following an overnight fast was substantially higher than when it was given in capsules with a light breakfast. As a result of these findings, the most appropriate technique for the oral delivery of EGCG in future clinical studies where EGCG is to be investigated as a potential bioactive nutraceutical in humans is to take it with water on an empty stomach [52]. Concomitant administration of bioenhancers such as ascorbic acid, fish oil, and piperine may act synergistically to improve EGCG bioavailability by inhibiting oxidation and suppressing glucuronidation, resulting in increased EGCG absorption [53, 54].

### 2.4. Ginkgo Special Extract

*Ginkgo biloba* is the sole surviving plant in the Ginkgo family, and it has been used to prevent neurological illnesses since antiquity [55, 56]. Active components in the standardized EGb 761 ginkgo extract include 24 percent ginkgo-flavone glycosides, 6 percent terpenoids, and 5–10 percent organic acids. Ginkgo's antioxidant qualities, vascular remodelling properties, and neurotransmitter-potentiating activities can be utilized to treat a variety of neurological diseases, including AD and depression [57]. Clinical trials in Germany by Kanowski and Hoerr [58] and the United States by Le Bars et al. [35] to test the efficacy of *Ginkgo biloba* on dementia has yielded positive findings (Table 1) in both 240 mg daily doses for 24 weeks and 120 mg daily dose for 26 weeks investigations. The research was extended for another 26 weeks; however, only 50 percent of EGb-treated patients and 38 percent of placebo-treated participants made it to the 52-week visit [36]. The active treatment outperformed the placebo in terms of improving patients' cognitive function and neuropsychiatric symptoms. The clinical significance of the pharmacological effects was demonstrated by the consistency of both primary and secondary outcomes, such as functional status, global evaluation, quality of life, and response rates. *Ginkgo biloba* extract appears to be well tolerated in the studies reviewed, without any significant differences between treatment and placebo, considering adverse effects and study withdrawals [58].

The article "Therapeutic Implications of Some Natural Products for Neuroimmune Diseases: A Narrative of Clinical Studies Review" was published in 2023. Journal: Evid Based Complement Alternat Med.

Johnson et al. conducted a clinical trial to investigate if the consumption of 240 mg of a ginkgo extract (EGb 761) per day for four weeks enhanced functional performance in MS patients. On measures of fatigue, symptom severity, and functionality, the ginkgo group had considerably more participants exhibiting improvement on four or more measures and less fatigues [33]. Despite the fact that ginkgo appeared to have therapeutic effects in some of the subjects, it is conceivable that the treatment duration was short. Furthermore, the individual therapeutic responses might vary. Thus, the result is that combining positive and negative responses in analyses may disguise or obfuscate some of the ginkgo's beneficial benefits [33, 34].

### 2.5. Ashwagandha *(Withania somnifera)*

From ancient times, *Withania somnifera* (WS), also known as ashwagandha, has been a significant plant in Ayurvedic and traditional medical systems [59]. The two main active components in ashwagandha are withaferin A and withanolide D, which have antioxidant, anti-inflammatory, immunomodulatory, anxiolytic, antidepressive, and neuroprotective properties [60, 61]. Because of these alleged healing effects, WS is widely used in Ayurvedic medicine, and it has been explored as a treatment for a variety of disease conditions including anxiety, inflammation, PD, and cognitive impairment [62]. *Withania somnifera* is also used as an immunological stimulant in individuals with low white blood cell counts and as an adaptogen for patients with fatigue, sleeplessness, and stress disorders [62, 63]. A study that looked at the effects of a Withania extract on calcium antagonism in the central nervous system shed some information on a possible anxiolytic mode of action. In this investigation by Grunze et al. [64], treatment with Withania extract caused extracellular calcium antagonism in neurons, counteracting excitement. Calcium excitation has been found to play a role in a variety of psychiatric diseases, including anxiety, so inhibiting calcium excitation should have an anxiolytic effect.

The article "Therapeutic Implications of Some Natural Products for Neuroimmune Diseases: A Narrative of Clinical Studies Review" was published in 2023. Journal: Evid Based Complement Alternat Med.

According to a clinical trial conducted by Langade et al. [29], Ashwagandha root extract (KSM 66 pill) of 300 mg twice daily dosage for a period of 10 weeks improved sleep parameters in individuals with insomnia and anxiety (Table 1). When compared to the placebo group, significant improvements in sleep quality and sleep metrics such as sleep onset latency (SOL), sleep efficiency (SE), Pittsburgh Sleep Quality Index (PSQI), and anxiety parameters such as the Hamilton Anxiety Rating Scale (HAM-A) were seen. In this context, oral administration of capsules containing Ashwagandha can be used as a potential anxiolytic agent (Table 1) [29].

### 2.6. *Centella asiatica* (*L*)

*Centella asiatica* is a herbaceous plant that can be found all throughout India, the Middle East, and Asia including Sri Lanka. The main bioactive compound of this plant is triterpene saponosides [65]. Furthermore, pharmacological studies have demonstrated that *C. asiatica* and its constituents, primarily asiaticoside and ursolic acid, exhibit a wide range of pharmacological actions, including memory boosting, sleep-inducing, anxiolytic, and antioxidant characteristics [66–68]. *C. asiatica* has also been shown to mitigate neurodegeneration and protect against oxidative stress-induced brain aging [66]. By these mechanisms, *C. asiatica* can exert neuroprotective effects against neuroimmune diseases such as AD, PD, depression, and anxiety [69–71].

A clinical study conducted by Jana et al. [30] to investigate the therapeutic efficacy of *C. asiatica* to treat psychiatric conditions such as generalized anxiety disorder found that oral administration of encapsulated 500 mg of *C. asiatica* plant extract twice daily after a meal for two months has been shown to effectively decrease stress anxiety-depression disorders (Table 1). No other anxiolytic drugs were given to the study subjects during the study period. The study found that after 60 days of treatment, the anxiety index, depression index, adjustment score, and attention level were significantly reduced, with no negative side effects. As a result, *C. asiatica* could be an alternative treatment agent for stress-related clinical illnesses [30].

### 2.7. Bacopa monnieri

*Bacopa monnieri,* often known as “Brahmi,” is a native plant that can be found in the Indian subcontinent, East Asia, and some parts of the United States. Its antianxiety, anti-inflammatory, memory boosting, and immunomodulatory properties are thought to be due to its antioxidant properties. Bacosides, one of its bioactive ingredients, have been proven to help with anxiety, depression, and cognitive impairment [72–74]. A clinical study of newly diagnosed AD patients found that taking a standardized extract of *Bacopa monnieri* (Bacognize®) 300 mg twice daily for six months improved their quality of life, enhanced their memory power, and reduced their irritability and insomnia, and some even reported positive changes in their family behavior (Table 1) [74].

The article "Therapeutic Implications of Some Natural Products for Neuroimmune Diseases: A Narrative of Clinical Studies Review" was published in 2023. Journal: Evid Based Complement Alternat Med.

It has been demonstrated that the natural product formula containing *B. monnieri* effectively increased minimental state examination (MMSE) scores in AD patients. A polyherbal compound's synergistic properties may aid in achieving beneficial results [42]. Sadhu et al. [43] reported that providing a polyherbal formula comprising *B. monnieri* at a dose of 500 mg over a 12-month period was effective in improving cognitive skills in individuals with senile dementia of Alzheimer's type (SDAT) when compared to the donepezil-treated group. Diminished inflammation and oxidative stress were indicated by reducing levels of homocysteine, C-reactive protein, superoxide dismutase, tumor necrosis factor-alpha (TNF-*α*), and glutathione peroxidase, in the SDAT patients treated with the test formulation when compared to the donepezil-treated group (Table 1). These results showed a protective effect of the test formulation in managing cognitive decline associated with the aging process [43]. A prior *in vivo* study showed that bacoside A encapsulation with nanoparticles might be a potential strategy to facilitate BBB penetration, thus enhancing therapeutic efficacy while treating neurodegenerative diseases. Therefore, *B. monnieri* may be a plausible therapeutic agent to enhance cognitive function in AD patients via a nanotechnological approach [42, 75].

### 2.8. Ginseng

Ginseng is a well-known herbal remedy that is widely used in traditional Chinese medicine as a tonic, restorative, and antiaging agent [76]. Ginsenosides are the main bioactive compounds in the plant, although there are also polysaccharides, triterpenoids, and flavonoids [77, 78]. Free radicals and oxidative stress may have a role in the development of fatigue in people with MS [79, 80]. Ginseng's antifatigue properties could be attributed to its antioxidant properties and ability to control GABAergic neurotransmissions [81].

Etemadifar et al. [37] conducted a pilot study to assess the efficacy and safety of ginseng in the treatment of fatigue in MS patients and found that the ginseng supplement was well tolerated with no significant adverse events after three months of daily administration of 500 mg of ginseng. The results showed that when ginseng was used instead of a placebo, the mean scores for the fatigue impact scale (MFIS) “physical” subscale improved significantly (*p*=0.046) [37]. Furthermore, as compared to the placebo group, most of the scores for the individual domains of the Multiple Sclerosis Quality of Life Questionnaire (MSQOL-54), including physical health, emotional well-being, energy, cognitive function, health distress, and quality of life, were significantly higher in the ginseng-treated group [37]. However, a human trial conducted by Kim et al. on the treatment of fatigue in 47 MS patients with progressively increasing doses of ginseng over a 6-week period found it to be safe but ineffective. This could be related to the study's short duration and the severity and stages of the disease [82]. Therefore, future clinical trials should be conducted over a considerable period of time to determine the efficacy of ginseng at various stages of the disease.

The article "Therapeutic Implications of Some Natural Products for Neuroimmune Diseases: A Narrative of Clinical Studies Review" was published in 2023. Journal: Evid Based Complement Alternat Med.

### 2.9. Cannabis

Cannabis plants are native to Central Asia that are grown all over the world [83]. D9-tetrahydrocannabinol (THC) is the main psychoactive component of cannabis, but other derivatives may have medicinal or synergistic properties. The most promising of these is cannabidiol (CBD), which is nonpsychoactive and may regulate THC's intoxication and/or memory effects. For its intoxicating qualities, high quantities of THC are preferred in the illegal market [83]. Therefore, standardized whole plant cannabis medical extracts (CBMEs) have recently been developed [84]. Inhalation and vaping are the most common ways to consume cannabis. Cannabinoids are rapidly absorbed into the bloodstream in this manner, with peak plasma THC concentrations reaching within minutes. Oral cannabis absorption and metabolism are unpredictable, and plasma concentrations are often sustained for longer periods of time (8–20 hours), resulting in inconsistent psychotropic effects [83].

With low degrees of intoxication, single case-crossover studies have shown that these CBMEs have the ability to diminish symptoms such as spasticity, pain, and spasms, in patients with MS [85]. Wade et al. conducted a trial using a whole plant extract including equal quantities (120 mg) of THC and CBD gave in a pump-action spray for the relief of MS symptoms. To mask the taste and appearance of CBME, all preparations included peppermint flavouring and colouring. Patients on an active treatment whose primary complaint was spasticity exhibited a substantial reduction (*p*=0.001) in contrast to placebo at the end of the study duration of six weeks. Patients with stable MS were given a two-week dose titration phase from 5 mg to a maximum of 25 mg of tetrahydrocannabinol daily, followed by a ten-week maintenance phase, according to Zajicek et al. [38]. After 12 weeks, the rate of relief from muscle stiffness was nearly twice as high with cannabis extract (CE) compared with place (Table 1). Even if the medical use of cannabis is clearly beneficial, it is important to be attentive in order to discover the potential for harm, particularly in relation to inhaled tobacco [83].

The article "Therapeutic Implications of Some Natural Products for Neuroimmune Diseases: A Narrative of Clinical Studies Review" was published in 2023. Journal: Evid Based Complement Alternat Med.

### 2.10. Future Prospects for Natural Product Clinical Research against Neuroimmune Diseases

Many factors should be considered in order to attain expected results from a natural product clinical trial. The findings of natural product clinical trials will be influenced by factors such as dose range, study period, number of patients enrolled, patient compliance, and clinical and biochemical response evaluations [86]. Adequate dose selection for confirmatory trials is still one of the most difficult problems to solve. The goal is to find the ideal target concentration that provides the most benefit with the least amount of side effects [87]. Acceptability of flavour, texture, and/or ease of swallowing capsules or tablets is critical for the participant's adherence to the study [88]. Future research should look into the mechanisms that explain why some people benefit from natural products while others do not so that treatment can be more useful and cost-effectively targeted to specific patients [33].

Novel drug-delivery systems, including liposomes, marinosomes, niosomes, and lipid-based systems, can improve bioavailability by increasing the rate of delivery and the ability to traverse lipid-rich biomembranes [89]. Phospholipid-based drug-delivery systems have been demonstrated to be effective and efficient in the delivery of herbal drugs [90]. Bioenhancers such as *Piper longum*, black pepper (*Piper nigrum),* long pepper (*P. longum*), and ginger (*Zingiber officinale*) are drug facilitators that enhance the activity of drug molecules which can be used in clinical studies to increase drug bioavailability across the membrane [91, 92]. Nanocarriers are being developed to overcome unmet drug-delivery hurdles and enable cross BBB. Extracellular vesicles have recently emerged as a natural carrier mechanism for therapeutic administration [93, 94]. Furthermore, gold nanoparticle-based drug-delivery systems are also capable of reaching the central nervous system [87]. It is worth noting that drug-delivery nanoparticles can either stimulate or inhibit the immune response, and they can reside in the body, so researchers must design appropriate nanodrugs, modify them according to disease characteristics, and conduct extensive immunotoxicology research before moving forward with clinical trials [95]. Natural product extracts may have a high concentration of constituents, and the combination of various active ingredients in extracts can provide synergistic effects, resulting in improved antioxidant and disease-modifying action [96, 97]. Identifying the compounds responsible for a particular biological action is challenging. For finding constituents that engage in synergistic effects, metabolomics and biochemometric methods are potential tools [98, 99]. Untargeted approaches to discovering synergistic molecular targets and unravelling synergistic mechanisms of action should be investigated [99]. Strategies to improve the outcome of natural product clinical studies are summarised in Figure 3. However, this review only focused on South Asian natural products, and due the discrepancies in clinical evaluation batteries/criteria in reviewed articles, we could not conduct a meta-analysis. We acknowledge this as a limitation in our study.

The article "Therapeutic Implications of Some Natural Products for Neuroimmune Diseases: A Narrative of Clinical Studies Review" was published in 2023. Journal: Evid Based Complement Alternat Med.

## 3. Conclusions

Positive results of clinical studies of natural products and their phytochemicals, such as curcumin, epigallocatechin-3-gallate (EGCG), ginkgo special extract, ashwagandha, *Centella asiatica, Bacopa monnieri*, ginseng, and cannabis against neuroimmune diseases, amply prove that they have therapeutic potential. One of the challenges that remain with their use is to maintain the stability of the unstable active ingredients of these natural products until they reach the target site. Inadequate dosages, poor aqueous solubility, and inadequate oral absorption via the oral route due to metabolism in the gastrointestinal tract and the inability to cross the BBB are the main considerations for natural products in clinical studies. Therefore, it is very important to evaluate the kinetic and physicochemical properties to develop such drugs and their delivery systems. The importance of multitarget combination therapies and the concept of synergy in the polyherbal formulation have risen to the fore. Future research should focus on identifying the combination of effects within complex mixtures, assuring a favourable outcome in natural product clinical studies. Chemical modification and encapsulation into nanoparticles may boost their efficacy and curtail systemic toxicity. Future studies are required to determine the correct techniques for natural products and their nanoformulations to convert them into probable drug candidates to treat neuroimmune diseases. The development of such nutraceuticals may pave the way toward novel therapeutic strategies to mitigate chronic neuroinflammation and overcome neuroimmune disorders.

The article "Therapeutic Implications of Some Natural Products for Neuroimmune Diseases: A Narrative of Clinical Studies Review" was published in 2023. Journal: Evid Based Complement Alternat Med.

## Figures and Tables

**Figure 1:** Summary of the review methodology.

**Figure 2:** Bidirectional communication between the nervous system and the immune system. Activated neurons release neuropeptides that activate inflammatory cells, and then various cytokines, chemokines, growth factors, leukotrienes, and prostaglandins are released from these inflammatory cells to act on nerve terminals. Substance P release from nerve terminals causes vasodilatation. IL-4 and IL-13 play a role to induce macrophages. Once induced, the macrophages produce various anti-inflammatory cytokines including IL-10, IL-13, and TGF-*β*, neurotrophic factors (insulin-like growth factor-1 (IGF-1)), brain-derived neurotrophic factor (BDNF), vascular endothelial growth factor, epidermal growth factor, and IL-1 receptor antagonist. Furthermore, macrophages play a role to block iNOS to reduce inflammation, protect cells, and maintain the stability of the environment in the body.

**Figure 3:** Strategies to improve the outcome of natural product clinical studies.

**Table 1:** Natural product clinical studies for neuroimmune diseases.

Natural product		Neuroimmune disease	Study design	Study participants	Dose	Duration	Assessment tool	Results	Conclusion	References
Ashwagandha	Ashwagandha root extract (KSM 66 capsule)	Anxiety disorder with insomnia	Randomized, double-blind parallel group, placebo-controlled study	80 participants	Ashwagandha root extracts 300 mg twice daily milk or water	Ten weeks	Sleep actigraphy (Respironics Philips) for assessment of sleep onset latency (SOL), total sleep time (TST), sleep efficiency (SE), and wake after sleep onset (WASO). , mental alertness on rising, sleep quality, Pittsburgh sleep quality index (PSQI), and Hamilton anxiety rating scale (HAM-A)	The sleep onset latency was improved in both test and placebo at five and 10 weeks. However, the SOL was significantly shorter (*p*, 0.019) after 10 weeks with test compared to placebo, significant improvement in SE scores and all other sleep parameters	Ashwagandha root extract contains natural compounds with sleep-inducing potential, well tolerated and improves sleep quality and sleep onset latency in patients with insomnia. It could be of potential use to improve sleep parameters in patients with insomnia and anxiety	[29]

*Centella asiatica* (CA)	The encapsulation contained 500 mg of the plant extract (CA)	Generalized anxiety disorder (GAD)	Open clinical trial	33 participants	500 mg/capsule, twice daily, after meal	Two months	Hamilton's brief psychiatric rating scale (BPRS)	CA not only significantly (*p* < 0.01) attenuated anxiety related disorders but it also significantly (*p* < 0.01) reduced stress phenomenon, and its correlated depression. CA further significantly (*p* < 0.01) improved the willingness for adjustment and cognition	Results indicated that *Centella asiatica* may be useful in the treatment of GAD and may be used as a promising anxiolytic agent .	[30]

Curcumin	Brainoil containing curcumin (600 mg), 100 mg of coenzyme Q10, 300 mg of *Bacopa monnieri*, 250 mg of *Withania somnifera*, and *Centella asiatica* (250 mg)	Amyotrophic lateral sclerosis (ALS	Double-blinded placebo-controlled study	42 participants	Curcumin oral supplementation (600 mg/day, group A received placebo for 3 months, then Brainoil for the following 3 months, group B took Brainoil for 6 months	Six months	Clinical evaluations and oxidative stress biomarkers, including oxidative protein products (AOPPs), ferric reducing ability (FRAP), total thiols (T-SH) and lactate	Reduction of AOPPs oxidative protein products (*p* < 0.01)Reduction of exercise lactate (*p* < 0.01)	Curcumin shows a slight slowdown in disease progression, improving aerobic metabolism and oxidative damage	[31]

Curcumin	Curcumin C3 Complex®	Alzheimer's disease	Randomized, double blind, placebo-controlled study	36 subjects	2 grams/day, or4 grams/day oral	Six months	Neuropsychiatric inventory (NPI), Alzheimer's disease cooperative study activities of daily living (ADCS-ADL), MMSE, plasma levels of A*β*1-40 and A*β*1-42, CSF levels of A*β*1-42, total tau	There were no differences between treatment groups in clinical or biomarker efficacy measures. The levels of native curcumin measured in plasma were low (7.32 ng/mL)	Curcumin C3 Complex® is ineffective in AD	[32]

*Ginkgo biloba* (GB)	Ginkgo special extract (EGb 761)	Multiple sclerosis (MS)	Double-blind, placebo-controlled, parallel group design	22 individuals	240 mg per day	One month	Depression (Center for Epidemiologic Studies of Depression Scale (CES-D)), anxiety (state-trait anxiety inventory (STAI)), fatigue (modified fatigue impact scale (MFIS)); symptom severity (symptom inventory (SI)) and functional performance (functional assessment of multiple sclerosis (FAMS))	The ginkgo group had significantly more individuals showing improvement on four or more measures with improvements associated with significantly larger effect sizes on measures of fatigue, symptom severity, and functionality. The ginkgo group also exhibited less fatigue at follow-up compared with the placebo group	This exploratory pilot study showed that no adverse events or side effects were reported and that ginkgo exerted the modest beneficial effects on select functional measures (e.g., fatigue) among some individuals with MS	[33]

*Ginkgo biloba* (GB)	Ginkgo biloba extract EGb 761	Multiple sclerosis (MS)	Randomized, double-blind, and placebo-controlled trial	43 individuals	240 mg per day	Three months	The three second version of the PASAT, the controlled oral word useful association test (COWAT), the symbol digit modalities test (SDMT), an adapted version of the useful field of view test (UFOV), Victoria version of the Stroop color and word test (stroop), MS quality of life index (MSQLI)	The GB group was faster than the placebo group on the color-word interference condition of the stroop test. Subjects who were more impaired at baseline experienced more improvement with GB (treatment ∗ baseline interaction, *F* = 8.10, *p*=0.008). No differences on the other neuropsychological tests. No serious drug related side effects occurred	Overall, GB did not show a statistically significant improvement in cognitive function. A treatment effect trend, limited to the stroop test, suggests that GB may have an effect on cognitive domains assessed by this test, such as susceptibility to interference and mental flexibility	[34]

*Ginkgo biloba*	*Ginkgo biloba* extract EGb 761	Dementia of the Alzheimer's type or multinfarct dementia	Double-blind, randomized, and placebo-controlled	222 patients	240 mg per day	Six months	SKT (Syndrom-Kurz test), clinical global impression of change (CGI), and Nurennerg gerento psychology observation scale	CGI and NAB, SKT scores showed mild improvement in *Ginko biloba* treated group	Treatment of *Ginkgo biloba* extract EGb 761 shows cognitive functions improvement in dementia patients.	[35]

*Ginkgo biloba*	*Ginkgo biloba* extract EGb 761	Dementia of the Alzheimer's type or multinfarct dementia	Randomized, double blind, placebo-controlled study	327 patients	120-mg dose	52-weeks	Alzheimer's disease assessment scale-cognitive subscale (ADASCog), geriatric evaluation by relative's rating instrument (GERRI), clinical global impression of change	Regarding the ADÄS-Cog, there was no significant change observed at end point for the EGb group, whereas the placebo group showed a significant worsening of 1.5 points (*p*=0.006). The mean treatment difference significantly favoured EGb (*p*=0.04). Considering the GERRI, mild improvement was observed for the EGb group, whereas the placebo group showed significant worsening (0.08 points; *p*=0.02), resulting in a statistically significant difference in favour of EGb (*p*=0.004)	In clinical terms, improvement on the ADAScog of 4 points may be equivalent to a 6-month delay in the progression of the disease	[36]

ginseng	Korean ginseng tablets	Multiple sclerosis (MS)	Randomized, double-blind, placebo-controlled pilot study	52. Female MS patients	250-mg	Three months	Modified fatigue impact scale (MFIS), Iranian version of the multiple sclerosis quality of life questionnaire (MSQOL-54)	Better effects for ginseng than the placebo as regards modified fatigue impact scale (MFIS) and multiple sclerosis quality of life questionnaire (MSQOL-54) (*p* ≤ 0.0001) after 3 months. No serious adverse events were observed during follow-up	This study indicates that 3-month ginseng treatment can reduce fatigue and has a significant positive effect on quality of life. Ginseng is probably a good candidate for the relief of MS-related fatigue	[37]

Cannabis	Cannabis sativaoral cannabis extract (CE)	Multiple sclerosis (MS)	Double blind, placebo controlled, phase III study	144 patients with stable MS	5 mg to a maximum of 25 mg of tetrahydrocannabinol daily	Three months	11 point CRS to evaluate perceived change in muscle stiffness, secondary outcome measures included further equivalent CRSs measuring perceived relief from body pain, muscle spasms, and sleep disturbance compared with pretreatment (at 4, 8, and 12 weeks)	The rate of relief from muscle stiffness after 12 weeks was almost twice as high with CE than with placebo	The study met its primary objective to demonstrate the superiority of CE over placebo in the treatment of muscle stiffness in MS. This was supported by results for secondary efficacy variables. Adverse events in participants treated with CE were consistent with the known side effects of cannabinoids	[38]

Cannabis	Cannabis-based whole plant medicinal extract (sativex)	Multiple sclerosis (MS)	A parallel group, double-blind, randomized, placebo-controlled study	160 patients	Equal amounts of delta-9-tetrahydrocannabinol (THC) and cannabidiol (CBD) at a dose of 2.5–120 mg of each daily	Two and half months	100 mm VAS for the primary target symptom, Barthel activities of daily living (ADL) index, Rivermead mobility index, adult memory and information processing battery test of attention adapted for patients with MS, adult memory and information processing battery test of attention adapted for patients with MS, the Beck depression inventory, the fatigue severity scale, the modified ash worth scale of spasticity	Following CBME the primary symptom score reduced. Spasticity VAS scores were significantly reduced by CBME (sativex) in comparison with placebo (*P*/0.001). There were no significant adverse effects on cognition or mood and intoxication was generally mild	The results of this study suggest that CBME (sativex) is an effective treatment for spasticity associated with MS. The use of gradual self-titration of the dose allowed most people to achieve benefit without unduly troublesome side effects	[39]

Epigallocatechin-gallate (EGCG)	Polyphenon E, a green tea extract containing 50% of the antioxidant epigallocatechin-gallate (EGCG)	Multiple sclerosis	PhI: single group futility study. PhII: parallel group randomized double-blind placebo-controlled study	23 participants	PhI: two capsules twice daily (200 mg of EGCG per capsule; total daily dose 800 mg), PhII : Polyphenon E or matching placebo capsules, same dose	Ph-1 -6 months, Ph2-12 months	PhI: (1) adverse events (AE); (2) futility: decrease in N-acetyl aspartate (NAA) from baseline to six months of 10% or more; (3) association between EGCG plasma levels and change in NAA. PhII: (1) AEs; (2) difference in the rate of change of NAA-levels over twelve months	The DSMB stopped the study because 5/7 participants had abnormal LFTs. Median time to onset of abnormal LFTs was 20 weeks	Class III evidence: 400 mg of EGCG twice a day is not futile at increasing brain NAA-levels. Class I evidence: some lots of EGCG have a high risk of hepatotoxicity	[40]

*Bacopa monnieri*	Bacopa monnieri standardized extract (Bacognize®)	Alzheimer's disease	Open label, prospective, uncontrolled, nonrandomized trial	39 patients	300 mg of Bacopa monnieri standardized extract (Bacognize®) orally twice a day	6 months	Minimental state examination scale (MMSES)	Statistically significant improvements in various components of MMSES including orientation of time, place & person, attention and in their language component in terms of reading, writing and comprehension, improvement in their quality of life, and decrease in the irritability and insomnia at the end of trial	Bacopa monnieri standardized extract (Bacognize® 300 mg twice a day orally) for 6 months results in improvement in some aspects of cognitive functions patients suffering from Alzheimer's disease	[41]

Combination of nutraceuticals based on *Bacopa monnieri*, L-theanine, *Crocus sativus*, copper, folate and vitamins of B and D group	Not applicable	Dementia, depression	Double bind, crossover designed trial versus placebo setting	30 elderly subjects	Treatment with a combination of nutraceuticals based on *Bacopa monnieri*, L-theanine, *Crocus sativus*, copper, folate and vitamins of B and D group	Two months	Minimental state examination (MMSE), perceived stress questionnaire (PSQ), and index and self-rating depression scale (SRDS)	MMSE and PSQ-index significantly improved in the active treatment arm, both versus baseline and versus the parallel arm. Both groups experienced a significant improving in the SRDS scores	Significant improvement of the cognitive functions tested with the MMSE, PSQ-index and SRDS score, after 2 months of combined therapy of nutraceuticals	[42]

Formulation containing extracts of *Bacopa monnieri* (whole plant), *Hippophae rhamnoides* (leaves and fruits), and *Dioscorea bulbifera* (bulbils)	Not applicable	Senile dementia of Alzheimer's type (SDAT)	A randomized double-blind placebo- and active-controlled clinical trial	109 healthy subjects and 123 SDAT patients	500 mg	Twelve months	Minimental state examination (MMSE) score, digital symbol substitution (DSS; subtest of the Wechsler adult intelligence scale-revised), immediate and delayed word recall (digital memory apparatus-medicaid systems, Chandigarh, India), attention span (attention span apparatus-medicaid systems, Chandigarh, India), functional activity questionnaire (FAQ), and depression (geriatric depression scale) scores	Improvements in various cognitive and neuropsychiatric measures like minimental state examination (MMSE) score, digital symbol substitution (DSS; subtest of the Wechsler adult intelligence scale—revised), immediate and delayed word recall, attention span, functional activity questionnaire (FAQ), and depression (geriatric depression scale) scores. This was accompanied by a reduction in inflammation and oxidative stress as determined by the measurement of various markers such as SOD, GPx, GSH, TBARS, IL-6, TNF-a, CRP, and homocysteine in the blood plasma	Administration of the test formulation for a period of 12 months was effective in improving cognitive functions in the SDAT patients. These findings suggest that the test formulation is a safe novel polyherbal drug product and has immense therapeutic potential for the management and treatment of neurodegenerative disorders	[43]

Nanocurcumin	Not applicable	Multiple sclerosis (MS)	Randomized, double-blind, placebo-controlled trial	50 patients with multiple sclerosis	Nanocurcumin	Six months	Gene expression levels of miRNAs, and miRNA-dependent targets, and also transcription factors and proinflammatory cytokines in blood samples	According to the results, a significant decrease in mRNA expression levels of miR145, miR-132, miR-16, STAT1 (*p*=0.0002), NF-*κ*B,AP-1, IL-1*β*, IL-6, IFN–*γ*, CCL2, CCL5, TNF-*α,* and significant increase in expression levels of miRNAs targets; Sox2, sirtuin-1, Foxp3, and PDCD1 was evident in nanocurcumin treated group compared with before treatment. The secretion levels of IFN–*γ*, CCL2, and CCL5. (*p*=0.0003) were reduced dramatically in test group compared with the placebo group	Nanocurcumin could decrease mRNA expression levels of proinflammatory cytokines and transcriptional factors and also secretion levels in MS patients. Therefore, nanocurcumin can be used as a potential for improvement of MS symptoms	[44]

The article "Therapeutic Implications of Some Natural Products for Neuroimmune Diseases: A Narrative of Clinical Studies Review" was published in 2023. Journal: Evid Based Complement Alternat Med.

## Data Availability

The data used to support the findings of this study are available from the corresponding author on request.

## Abbreviations

CNS: Central nervous system
AD: Alzheimer's disease
PD: Parkinson's disease
ALS: Amyotrophic lateral sclerosis
HD: Huntington's disease
MS: Multiple sclerosis
BBB: Blood-brain barrier
BNB: Blood-nerve barrier
FDA: United States Food and Drug Administration
NaB: Sodium benzoate
EG: Epicatechin gallate
EGCG: Epigallocatechin-3-gallate
MMSE: Minimental state examination
SDAT: Senile dementia of Alzheimer's type
THC: D9-tetrahydrocannabinol
CBME: Cannabis medical extracts.
